The article "Anti-Tuberculosis Drug Induced Hepatotoxicity among TB/HIV Co-Infected Patients at Jimma University Hospital, Ethiopia: Nested Case-Control Study" was published in 2013. Journal: PLoS One.

# Anti-Tuberculosis Drug Induced Hepatotoxicity among TB/HIV Co-Infected Patients at Jimma University Hospital, Ethiopia: Nested Case-Control Study

**DOI:** 10.1371/journal.pone.0064622

**Published:** 2013-05-16

**Authors:** Alima Hassen Ali, Tefera Belachew, Alemeshet Yami, Wubeante Yenet Ayen

**Affiliations:** 1 School of Pharmacy, Jimma University, Jimma, Ethiopia; 2 Department of Population and Family Health, Jimma University, Jimma, Ethiopia; 3 Department of Internal Medicine, Jimma University, Jimma, Ethiopia; Barcelona University Hospital, Spain

## Abstract

**Background:**

This study was carried out to determine the incidence and predictors of anti-tuberculosis drug induced hepatotoxicity among TB/HIV co-infected patients at Jimma University Hospital, Ethiopia.

**Methods/Principal Findings:**

A nested case-control study was conducted by reviewing charts of all TB/HIV co-infected patients who commenced anti-TB treatment from January 2008 to December 2011 at Jimma University Hospital. Patients who had developed hepatotoxicity after at least 5 days of standard doses of anti-TB drug therapy were labeled as “cases” and those without hepatotoxicity were “controls”. Each case with anti-TB drug induced hepatotoxicity was compared with 3 controls selected randomly from the cohort. From a cohort of 296 TB/HIV co-infected patients 8 were excluded from the study as the causality between anti-TB drugs and hepatotoxicity was not confirmed, 33 had developed hepatotoxicity. On bivariate logistic regression analysis, body mass index (BMI) <18.5 Kg/m^2^ [P = 0.01; OR (95%CI): 3.6 (1.4–9.5)], disseminated pulmonary TB [P = 0.00; OR (95%CI): 5.6 (2.2–14.6)], CD4 count ≤50 [P = 0.016; OR (95%CI): 3.6(1.27–10.23)] and WHO stage 4 [P = 0.004, OR (95%CI): 3.8 (1.68–8.77)] were significantly associated with anti-TB drug induced hepatotoxicity. Predictor variables with p-value <0.05 by bivariate analysis were analyzed using multivariable logistic regression analysis and identified disseminated pulmonary TB [P = 0.001; AOR (95%CI)  = 5.6 (2.1–15.0)] and BMI <18.5 [P = 0.014; AOR (95%CI)  = 3.6 (1.3–10.1)] as independent predictors of anti-TB drug induced hepatotoxicity.

**Conclusions:**

The incidence of anti-TB drug induced hepatotoxicity was 11.5%. The results suggest that in the presence of disseminated pulmonary TB and/or BMI <18.5 Kg/m^2^, TB/HIV co-infected patients should be closely followed for the occurrence of hepatotoxicity during the intensive phase of TB treatment to prevent morbidity and mortality.

## Introduction

The human immunodeficiency virus (HIV) epidemic led to major upsurge in tuberculosis (TB) cases and TB mortality in many countries specially southern and eastern Africa. The World Health Organization (WHO) has classified Ethiopia as 7^th^ among the 22 high burden countries with TB/HIV co-infection in the world and that reported lower rate of treatment success. HIV infection significantly increases the risk of progression from latent to active TB disease. According to WHO reports, globally there were over one in ten of the 9 million people who developed TB each year, which is equivalent to 1.1 million new TB cases among people living with HIV in 2010 [1].

The article "Anti-Tuberculosis Drug Induced Hepatotoxicity among TB/HIV Co-Infected Patients at Jimma University Hospital, Ethiopia: Nested Case-Control Study" was published in 2013. Journal: PLoS One.

Active TB disease requires prompt initiation of TB treatment. The treatment of active TB disease in HIV infected patients should follow the general principles for individuals without HIV. Treatment of drug susceptible TB disease should include a standard regimen that consists of first line drugs isoniazid, rifampicin, pyrazinamide, ethambutol or streptomycin given for 2 months, followed by isoniazid and rifampicin/ethambutol for 4 to 7 months [2].

All HIV positive patients with active TB disease should start antiretroviral treatment (ART). However, there is approach that we might need to start treating the TB first and wait on ART, if there are significant drug interactions between anti-TB drugs and ART. Studies showed that ART can reduce the risk of death in patients co-infected with TB/HIV [3], [4]. The latest policy guidance from WHO recommends that ART should be provided to all TB/HIV co-infected patients, irrespective of their CD4 cell count (and to all people living with HIV/AIDS with a CD4 cell count less than 350). However, concomitant use of anti-TB and antiretroviral (ARV) drugs is complicated by adherence challenge of pill burden, drug-drug interaction, overlapping adverse effects, one of the serious adverse effect is hepatotoxicity [5].

Anti-TB drug induced hepatotoxicity, which is a common serious adverse drug reaction, is one of the most challenging clinical problems and main cause of treatment interruption during TB treatment course that causes hospitalization and life threatening event [6]–[8]. Among the first line anti-TB drugs, pyrazinamide, isoniazid and rifampicin have all been associated with hepatotoxicity and the risk is enhanced when these drugs are used in combination [9]. Different studies reported that 1–31% of TB patients experience drug related hepatotoxicity following TB treatment [10]–[14].

Identification of patients at increased risk for anti-TB drugs induced hepatotoxicity is important because hepatotoxicity can cause economical burden, prolong duration of illness, morbidity and mortality, and may require modification of dosage regimen. Although there are considerable number of HIV infected patients on TB treatment at Jimma University Hospital (JUH), to-date there have been no published studies identifying predictors for the development of anti-TB drug induced hepatotoxicity among TB/HIV co-infected patients. Besides there are no studies that showed the incidence of anti-TB drug induced hepatotoxicity among TB/HIV co-infected patients in the study area. Therefore, given the paucity of studies on anti-TB drugs and hepatotoxicity, the primary objective of this study is in order to determine incidence and assess possible risk factors for developing anti-TB drugs induced hepatotoxicity among TB/HIV co-infected patients admitted to JUH, Ethiopia. Therefore, identifying risk factors might help prevent or monitoring patients more closely and it might decrease the burden related to hepatotoxicity.

The article "Anti-Tuberculosis Drug Induced Hepatotoxicity among TB/HIV Co-Infected Patients at Jimma University Hospital, Ethiopia: Nested Case-Control Study" was published in 2013. Journal: PLoS One.

## Methods

### Study Design

A retrospective nested case-control study of TB/HIV co-infected patients was conducted in order to examine the incidence and predictors of anti-TB drugs induced hepatotoxicity.

### Setting and Period

This study was conducted from February to May 2012 at TB/HIV care clinic of Jimma University Hospital. Jimma University Hospital is the only teaching and referral hospital located in Jimma Town, in the Southwestern part of Ethiopia. It provides services for approximately 9000 inpatient and 80,000 outpatient attendances a year from the catchment population of about 15 million people. It has bed capacity of 450 and a total of more than 750 staff, both supportive and professional. TB/HIV care clinic is one of the chronic follow-up clinics of the hospital providing services from Monday to Friday.

### Study Population

Data was obtained from patient database, which is computerized registry of HIV patients. In TB/HIV care clinic, a total of 9,809 HIV infected individuals (including TB/HIV co-infected patients) were enrolled, out of which 3,519 commenced ART till study period. From a computerized registry of HIV patients, a cohort of 296 TB/HIV co-infected patients those who commenced anti-TB drugs from January1, 2008 to December 31, 2011 were included in the study. Patients with anti-TB drug induced hepatotoxicity (cases) using biochemical criteria and clinical judgment, who developed 5 days after start of standardized anti-TB drugs, were identified as cases and each case was matched with three controls (without hepatotoxicity) selected randomly from cohorts of 296 TB/HIV co-infected patients. The patients (inpatients and/or outpatients) fulfilled the following inclusion criteria: Patients who have baseline and follow-up liver enzyme tests and showed completely normal findings on alanine aminotransferase (ALT) and aspartate aminotransferase (AST) at the beginning of treatment; patients who received standard doses of anti-TB drugs for at least five days prior to the development of hepatotoxicity. Exclusion criteria: Patients receiving a higher dosage of anti-TB drugs than the recommended dosage according to body weight.

The article "Anti-Tuberculosis Drug Induced Hepatotoxicity among TB/HIV Co-Infected Patients at Jimma University Hospital, Ethiopia: Nested Case-Control Study" was published in 2013. Journal: PLoS One.

### Treatment protocol/follow-up

All TB/HIV co-infected patients are evaluated by a multidisciplinary team of internists, medical residents, senior medical students, clinical pharmacists, laboratory technologists and general nurses at baseline and throughout their treatment. They have regular monitoring of liver function tests, hemoglobin level, renal function test, and CD4 count before and during the course of treatment as per national TB/HIV treatment guidelines. In addition, body weight, adherence to medication, adverse drug reaction and other relevant parameters are also monitored during each visit. Patients with evidence of complications of disease and/or adverse drug reactions get frequent check-ups. Case definition of TB includes those new patients who have smear-positive Pulmonary TB and those who seriously ill patients with smear-negative Pulmonary and Extra-pulmonary TB (category I). Hence, newly diagnosed TB case (recurrence or relapse excluded) was classified in the medical files in terms of its clinical type as pulmonary, extra pulmonary or disseminated pulmonary TB. TB treatment was given based on National Standard Treatment Guideline for hospitals, Ethiopia. The treatment (empiric) consists of 8 weeks with fixed dose combination of rifampicin, isoniazid, pyrazinamide and ethambutol (RHZE as 150/75/400/275mg mg tablet) during the intensive phase followed by rifampicin and isoniazid (RH as 300/150mg) for 4 months or ethambutol and isoniazid (EH as 400/150mg) for 6 months during continuous phase depending on category of TB. Everyone receives the same regimen but different doses based on body weight. Patients were given directly observed treatment short course (DOTS) by medical staffs of the clinic. Daily doses are calculated based on body weight.

### Diagnosis of anti-TB drug induced hepatotoxicity

Clinician judgment and/or biochemical criteria (increased level of liver enzymes) guided the decision to anti-TB drugs induced hepatotoxicity and include presence of one of the following criteria.

- A rise to ≥3 fold the upper limit normal (ULN) of ALT and/or AST.
- Any increase above pre-treatment values together with anorexia, nausea, vomiting or jaundice.
- Normalization of liver enzymes level and resolution of signs and symptoms of hepatotoxicity after withdrawal of all anti-TB drugs.

Normal maximum value in the laboratory is 40 IU/L for ALT and 37 IU/L for AST, which is same cut-offs for men and women. The degree of severity of hepatotoxicity was evaluated based on WHO Toxicity Classification Standards [11]. Mild hepatotoxicity is defined as AST and/or ALT elevations of <3 fold the ULN (<121 IU/L); moderate hepatotoxicity as elevations of 3–5 fold the ULN (121–200 IU/L); severe hepatotoxicity as elevations 5–10 times (201–400 IU/L) and very severe hepatotoxicity >10 times the ULN (>400 IU/L) or more than 250 IU/L with symptom of fulminant hepatitis as evidenced by jaundice and/or lethargy.

The article "Anti-Tuberculosis Drug Induced Hepatotoxicity among TB/HIV Co-Infected Patients at Jimma University Hospital, Ethiopia: Nested Case-Control Study" was published in 2013. Journal: PLoS One.

### Data Analysis

For the purpose of this study, the risk factors considered were age group (young versus older), gender, CD4 count, WHO clinical stage of HIV/AIDS, body weight/body mass index, type of TB, ART regimen and other co-administered medications. The dependent variable was the occurrence of anti-TB drugs induced hepatotoxicity. Categorical variables were presented in frequencies and percentages, whereas numerical variables were expressed in means and standard deviations. The various risk factors in the study population were analyzed using the independent *t*-test to compare means of continuous variables and chi-square test for categorical variables to evaluate their association with the development of hepatotoxicity at a significance level of p-value <0.05 for rejection of the null hypothesis of absence of association between the variables. The variables that presented associations with the outcome after bivariate analyses were entered into multivariate logistic regression model to identify independent predictors of anti-TB drugs induced hepatotoxicity. The probabilities of developing hepatotoxicity with duration of anti-TB drugs treatment were estimated by Kaplan Meier methods and log-rank test was used to determine statistically significant association. Statistical Package for the Social Sciences, version 16.0 (SPSS Inc. Michigan, USA) was used for analysis of data.

### Ethics Statement

Approval for conducting study was obtained from institutional review board, Jimma University. Patient consent was not obtained due to retrospective nature of the present study and any personally identifiable information was not collected and made available to maintain confidentiality.

## Results

Forty-one of 296 (13.85%) TB/HIV co-infected patients, who had anti-TB drugs, were identified as having evidence of increased liver enzyme levels. Among 41 patients, 33 were eligible for definite diagnosis of anti-TB drugs induced hepatotoxicity. The remaining 8 patients were excluded from the study as there was no clear causality relationship between anti-TB drugs administration and hepatotoxicity. The actual attribute to the increased liver enzymes in the 8 patients remains unknown by the authors as all drugs including anti-TB drugs, ARVs and co-trimoxazole were discontinued for all of 8 patients until the normalization of liver function tests in which the causative agent was not ruled out as medications stopped altogether. In the study population, the prevalence of anti-TB drug induced hepatotoxicity was 11.5% (33/288). Basic demographic and clinical characteristics of the patients are shown in Table 1.

The article "Anti-Tuberculosis Drug Induced Hepatotoxicity among TB/HIV Co-Infected Patients at Jimma University Hospital, Ethiopia: Nested Case-Control Study" was published in 2013. Journal: PLoS One.

**Table 1:** Demographic and clinical characteristics of 132 TB/HIV co-infected patients.

Variables	Cases (N = 33)	Controls (N = 99)
**Sex**		
Female	17 (51.5%)	53 (53.5%)
Male	16 (48.5%)	46 (46.5%)
**Age** (Mean ± SD)		
	32.5 [±8.6]	32.6 [± 8.2]
**CD4 cell count**		
≤50	14 (42.4%)	17 (17.2%)
51–100	7 (21.2%)	23 (23.2%)
101–200	4 (12.2%)	24 (24.2%)
>200	8 (24.2%)	35 (35.4%)
**Type of TB**		
Pulmonary	14 (42.4%)	63 (63.6%)
Extra pulmonary	4 (12.1%)	24 (24.2%)
Disseminated pulmonary	15 (45.5%)	12 (12.1%)
**Body mass index**		
<18.5	27 (81.8%)	55 (55.6%)
>18.5	6 (18.2%)	44 (44.4%)
**WHO stage**		
Stage 3	12 (36.4%)	68 (68.7%)
Stage 4	21 (63.6%)	31 (31.3%)
**ART**		
Yes	16 (48.5%)	67 (67.7%)
No	17 (51.5%)	32 (32.3%)
**ART regimen**		
NVP based regimen	6 (18.2%)	18 (18.2%)
EFV based regimen	10 (30.3%)	49 (49.5%)
**Co-trimoxazole**		
Yes	27 (81.8%)	75 (75.8%)
No	6 (18.2%)	24 (24.2%)
**Fluconazole**		
Yes	6 (18.2%)	7 (7.1%)
No	27 (81.8%)	92 (92.9%)

### General characteristics of study participants

There were 17 female patients (51.5%) among cases who had anti-TB drug induced hepatotoxicity and 53 (53.5%) among the control group. The mean age for cases and controls were 32.1 [±8.5] and 32.6 [±8.14] years, respectively, and ranged from 17 to 67 years of age (Table 1).

Of the total study participants, 82 (62.1%) had body mass index (BMI) <18.5 Kg/m^2^. Seventy seven (58.3%, N = 132) of all the study participants had pulmonary tuberculosis (PTB), 28 (21.2%, N = 132) had extra pulmonary tuberculosis (EPTB), while the remaining 27 (20.5%, N = 132) had disseminated pulmonary tuberculosis. The mean CD4 count was 116.9 [±116.4] and 188.7 [±169.9] for cases and controls, respectively. Twenty one (63.6%) and 31 (31.3%) were in WHO stage 4 from cases and control groups, respectively (Table 1).

Except 2 patients who were on 2HRZES/1HRZE/5HRE, all were on 2HRZE/4RH or 2HRZE/6HE anti-TB regimen. Eighty-three (62.9%, N = 132) of all study participants have been on ART (16 cases and 67 controls) before TB treatment, 22 (24.2%) were on ART for 325.5 (±42.4) mean days when anti-TB drug was started. The remaining 49 commenced ART after the diagnosis of TB and have been on anti-TB drug for mean of 39.4 (±30.5) days before initiation of ART. Most of patients, that is 27 (81.8%) from cases and 75 (75.7%) from control group were on cotrimoxazole prophylaxis, whereas only 6 (18.2%) from cases and 7 (7.1%) from control group were on fluconazole prophylaxis.

The article "Anti-Tuberculosis Drug Induced Hepatotoxicity among TB/HIV Co-Infected Patients at Jimma University Hospital, Ethiopia: Nested Case-Control Study" was published in 2013. Journal: PLoS One.

### Clinical and biochemical spectrum of anti-TB drugs induced hepatotoxicity

The time interval from initiation of ant-TB drugs to the onset of hepatotoxicity ranged from 8 to 90 days with a mean of 26 [±11.6] days. Most (93.9%) of the cases occurred during the first 6 weeks. AST and ALT in anti-TB drug induced hepatotoxicity patients ranged from 104 to 553 IU/L [mean of 220.8 [±114.2]] and 162.1 to 407.5 IU/L [mean of 182.6 [±75.6]], respectively (Table 2). Symptoms shown by all cases were gastrointestinal manifestations like nausea, vomiting, abdominal discomfort, anorexia, and/or jaundice. Severity of hepatotoxicity classified based on the level of biochemical derangement according to WHO adverse drug reaction grading system showed that very severe hepatotoxicity observed in 8 patients (24.2%, N = 33) while severe (grade 3) hepatotoxicity was found to be 7 (21.2%) (Table 3).

**Table 2:** Changes in liver function tests and clinical presentation of 33 TB/HIV co-infected patients who developed anti-TB drugs induced hepatotoxicity.

Variables	Measurements/Observations	No. of cases (%) (N = 33)
ALT	<3 times ULN (<121IU/L) with Jaundice	2 (6.1%)
	3–5 times ULN (121–200 IU/L)	24 (72.7%)
	5–10 times ULN (201–400 IU/L)	6 (18.2%)
	>10 times ULN (>400 IU/L)	1 (3.0%)
AST	<3 times ULN (<121 IU/L) with Jaundice	2 (6.1%)
	3–5 times ULN (121–200 IU/L)	16 (48.5%)
	5–10 times ULN (201–400IU/L)	11 (33.3%)
	>10 times ULN (>400 IU/L)	4 (12.1%)
ALT	Mean ± SD	182±75.6
AST	Mean ± SD	220±114.2
Clinical presentations	Jaundice and/or lethargy	13 (39.4%)
	Nausea, anorexia, or vomiting	25 (75.7%)

**Table 3:** Degree of severity of anti-TB drug induced hepatotoxicity, according to the WHO classification of drug toxicity.

Severity	Liver enzyme level	No. of cases (%) (N = 33)
Moderate	<5 times ULN (<200 IU/L)	18 (54.5%)
Severe	5–10 times ULN (201–400 IU/L)	7 (21.2%)
Very severe	>10 times ULN (>400 IU/L)	4 (12.1%)
	≥5 times ULN and Jaundice and/or lethargy	4 (12.1%)

### Factors associated with anti-TB drug induced hepatotoxicity

Age was categorized into younger (<35 years) and older (≥35 years) age groups and there was no difference between cases and controls between these age groups, and no correlation was found between age groups and incidence of anti-TB drugs induced hepatotoxicity. Nutritional status (as assessed by body mass index) of study participants seems poor (mean BMI <18.5 kg/m^2^). Cases were more likely to have malnutrition as compared to controls, 27 (81.8%) *vs.* 55 (55.6%), respectively; (P = 0.01). The mean BMI was significantly lower among cases as compared to controls, 15.51±2.91 kg/m^2^ *vs.* 18.46±2.42 kg/m^2^, respectively. Percent of patients with disseminated pulmonary TB was higher in the cases group, 15 (45.5%, N = 33) while in the controls group the number of disseminated pulmonary TB was 12 (12.1%, N = 99) (P = 0.001). Cases were also more likely to have lower CD4 count as compared to controls; 14 (42.4%, N = 33) of cases and 17 (17.2%, N = 99) of controls had CD4 count less than 50 (P = 0.016). Majority of cases, 20 (60.6%) were in WHO clinical stage 4 of HIV/AIDS; (P = 0.001). Therefore; BMI <18.5 kg/m^2^, disseminated pulmonary TB, lower CD4 count (≤50) and WHO clinical stage 4 of HIV/AIDS were significantly associated with anti-TB drug induced hepatotoxicity from bivariate model analysis (Table 4).

The article "Anti-Tuberculosis Drug Induced Hepatotoxicity among TB/HIV Co-Infected Patients at Jimma University Hospital, Ethiopia: Nested Case-Control Study" was published in 2013. Journal: PLoS One.

**Table 4:** Bivariate analyses of factors associated with anti-TB drug-induced hepatotoxicity.

Variables	Case (N = 33)	Control (N = 99)	COR (95% CI)	P
**Sex**				
Male	16	46	1.0	
Female	17	53	0.9 (0.4–2.0)	0.840
**Age**				
>35	9	33	1.0	
≤35	24	66	1.3 (0.5–3.2)	0.518
**BMI**				
≥18.5 Kg/m^2^	6	44	1.0	
<18.5 Kg/m^2^	27	55	3.6 (1.4–9.5)	0.010
**Type of TB**				
Pulmonary	14	63	1.0	
Extra pulmonary	4	24	0. 8 (0.2–2.5)	0.640
Disseminated pulmonary	15	12	5.6 (2.2–14.6)	0.000
**WHO stage**				
Stage 3	13	68	1.0	
Stage 4	20	31	3.8 (1.7–8.8)	0.004
**CD4 count**				
<50	14	17	3.6 (1.3–10.2)	0.016
50–100	7	23	1.3 (0.4–4.2)	0.623
101–200	4	24	0.9 (0.2–2.7)	0.636
>200	8	35	1.	
**On ART**				
Yes	16	67	0.4 (0.2–1.1)	0.051
No	17	32	1.0	
**ART regimen**				
NVP based regimen	6	18	0.9 (0.5–1.3)	0.76
EFV based regimen	10	49	1.0	
**Cotrimoxazole**				
Yes	27	75	1.4 (0.5–3.9)	0.473
No	6	24	1.0	
**Fluconazole**				
Yes	6	7	0.3 (0.1–1.1)	0.073
No	27	92	1.0	

COR: Crude Odds Ratio, BMI: Body mass index; NVP: nevirapine; EFV: efavirenz.

Multivariable logistic regression analysis was used to identify factors that are independently associated with the development of anti-TB drugs induced hepatotoxicity. All variables with P<0.05 in the bivariate model were included in the adjusted model using Backward Stepwise-Likelihood Ratio method. The analyses showed that the presence of disseminated pulmonary TB [AOR (95%CI)  = 5.6 (2.1–15.0); P = 0.001] and malnutrition i.e. BMI <18.5 Kg/m^2^ [AOR (95%CI)  = 3.6 (1.3–10.1); P = 0.014] were independent predictors in the development of anti-TB drugs induced hepatotoxicity in TB/HIV co-infected patients (Table 5).

**Table 5:** Multivariate regression analysis of factors associated with (or predictive factors of) anti-TB drug induced hepatotoxicity.

Variables	Case (N = 33)	Control (N = 99)	COR (95% CI)	P	AOR (95%CI)	P
**BMI**						
≥18.5	6	44	1.0			
<18.5	27	55	3.6 (1.4–9.5)	0.010	3.6 (1.3–10.1)	0.014
**Type of TB**						
Pulmonary	14	63	1.0			
Extra pulmonary	4	24	0. 8 (0.2–2.5)	0.640	0.7 (0.2–2.5)	0.621
Diss. pulmonary	15	12	5.6 (2.2–14.6)	0.001	5.6 (2.1–15)	0.001
**WHO stage**						
Stage 3	13	68	1.0			
Stage 4	20	31	3.8 (1.7 – 8.8)	0.001	2.4 (0.7–7.8)	0.120
**CD4 count**						
<50	13	17	3.6 (1.3 – 10.2)	0.016	2.3 (0.7–7.5)	0.160
50–100	7	23	1.3 (0.4 – 4.2)	0.623	1.6 (0.5–5.9)	0.450
101–200	5	24	0.9 (0.2 – 2.7)	0.636	0.8 (0.2–3.1)	0.710
>200	8	35	1.0			

AOR: Adjusted Odds Ratio; CI: Confidence interval; Diss.: Disseminated.

The article "Anti-Tuberculosis Drug Induced Hepatotoxicity among TB/HIV Co-Infected Patients at Jimma University Hospital, Ethiopia: Nested Case-Control Study" was published in 2013. Journal: PLoS One.

Mean time to onset of anti-TB drugs induced hepatotoxicity were lower among patients with disseminated pulmonary TB as compared to pulmonary TB and extra pulmonary TB (EPTB); 23.8[±5], 33.3[±13] and 36.5[±9], respectively (P = 0.253) (Figure 1). Kaplan Meier analysis shows that patient with lower BMI (<18.5 kg/m^2^) were likely to develop hepatotoxicity within 27.3[±6.5] mean days while those patients with BMI ≥18.5 kg/m^2^were likely to develop hepatotoxicity in 41[±20.7] mean days of commencing ant-TB drugs (P = 0.202) (Figure 2).

**Figure 1:** Duration of patients stay on anti-TB drugs before the occurrence of hepatotoxicity by the type of TB.

**Figure 2:** Duration of patients stay on anti-TB drugs before the occurrence of hepatotoxicity by BMI.

## Discussion

In the present study several important findings were observed and the incidence of anti-TB drugs induced hepatotoxicity among TB/HIV co-infected patients was 11.5%, which was in variance with other finding (30.0%) reported by Getnet Y. et al. [15]. This could be explained by the fact that the present study did not include the effect of ART induced hepatotoxicity as well as the retrospective nature of the study that can result in low incidence rate due to poor documentation and record keeping. However, the current finding is in consistent with the results of other studies [16]–[19].

In the present study pattern of alteration of liver enzymes was evaluated. The mean time elapsed between initiation of anti-TB drugs and elevation of aminotransferases was 26 [±11.6] days. Most, 31 (93.9%) of the cases occurred during the first 6 weeks. Different studies reported comparable findings, which showed that anti-TB drugs induced hepatotoxicity more commonly observed in the first 8 weeks. The median time until the development of hepatotoxicity in TB/HIV co-infected patients was 14 days (range 4–60) as previous report by Pukenyte E, et al. [20]. Study conducted in Brazil on hepatotoxicity due to anti-TB drugs in TB/HIV co-infected patients showed that more than 90% of hepatotoxicity occurred within the first 6 weeks of TB treatment [21]. The current finding is also in agreement with findings by Shakya R, et al. who reported that the time interval for onset of hepatotoxicity after initiation of therapy was 12–60 days [17]. Similarly, WV Senaratne, et al. reported that among 74 (9.5%) patients, who developed anti-TB drugs induced hepatotoxicity, the majority (58%) occurred within the first 2 weeks of the intensive phase treatment [18]. This could significantly affect the TB treatment, which potentially leads to unsuccessful treatment outcomes and the prolongation of intensive treatment phase. It emphasizes the importance of close and more frequent monitoring of patients in the intensive phase of anti-TB drugs therapy.

The article "Anti-Tuberculosis Drug Induced Hepatotoxicity among TB/HIV Co-Infected Patients at Jimma University Hospital, Ethiopia: Nested Case-Control Study" was published in 2013. Journal: PLoS One.

The finding of this study indicated that very severe (grade 4) hepatotoxicity accounts 8 (24.4%) of all anti-TB drugs induced hepatotoxicity while severe (grade 3) hepatotoxicity was found to be 7 (21.2%). Pukenyte E et al found that 10.7% incidence of severe hepatotoxicity in HIV infected patients who were on anti-TB treatment [20]. In the present study, all patients were hospitalized and required frequent monitoring of liver enzyme level and vital signs. From clinical and biochemical monitoring, abnormalities of liver functions and symptoms shown by patients suggested discontinuing of anti-TB drugs and all anti-TB drugs were temporarily discontinued following hepatotoxicity. Within 7 to 24 days of cessation of drugs, ALT and AST levels returned to normal and symptoms resolved. This proves that all signs and symptoms presented by the patients are related to the administration of anti-TB drugs and the finding is in consistent with other reports [17], [19]. Upon restart or re-challenge of anti-TB drugs, there were dose reduction and/or regimen change for 22 patients. All patients were under close supervision and monitoring of laboratory and vital signs until medication is tolerated. It was showed that upon restarting of anti-TB drugs, five patients developed hepatotoxicity while the rest tolerated the drugs with minimal elevation of liver enzymes and no clinical symptoms were observed. Patients who showed elevation in aminotransferases (3 to 5× ULN) upon restart and asymptomatic were continuing their anti-TB drugs, but under strict observation and frequent checkups. Fortunately, it was observed that their liver enzyme levels normalized within a few days upon continued treatment.

Disseminated pulmonary TB, lower BMI, WHO clinical stage 4 and lower CD4 count were found to be associated with increased risk of developing anti-TB drugs induced hepatotoxicity on bivariate analyses. However, on multivariable binary logistic regression analyses, disseminated TB and lower BMI (<18.5 Kg/m^2^) were found to be significant predictors in the development of anti-TB drugs induced hepatotoxicity.

The article "Anti-Tuberculosis Drug Induced Hepatotoxicity among TB/HIV Co-Infected Patients at Jimma University Hospital, Ethiopia: Nested Case-Control Study" was published in 2013. Journal: PLoS One.

Disseminated pulmonary TB was found to be one of the independent predictor of hepatotoxicity in the present study. This increased risk of developing hepatotoxicity in patients with disseminated pulmonary TB suggests that this group of patients may have subclinical hepatic involvement, which predisposes them to develop anti-TB drugs induced hepatotoxicity. There are reports indicating that organ (liver) involvement/extent of TB disease has been incriminated as positive predictor of drug induced hepatotoxicity, whereas extra pulmonary TB may not necessarily involve liver [22]–[24]. This implies a regular monitoring of liver function tests is mandatory in this group of patients.

Malnutrition status (assessed by body mass index, <18.5 kg/m^2^, [25]) is suggested as a risk factor for anti-TB drugs induced hepatotoxicity, a finding which is in consistent with other [18], [26]. The possible explanation of anti-TB drugs induced hepatotoxicity in malnutrition may be due to depletion of glutathione stores, which makes patients more vulnerable to oxidative injuries, and the slower pace at which the liver metabolize drugs [19], [24], [27].

In previous study conducted in Ethiopian HIV positive and negative TB patients, the development of anti-TB drugs induced hepatotoxicity had a significant association with decrement in the immune status of the patients as measured by the CD4 count [10]. Patients with CD4 count less than 50 were at increased risk of anti-TB drugs induced hepatotoxicity. However, in the present study, CD4 count (<50) was identified as risk factor on the bivariate analyses, the association disappeared on the adjusted model indicating that CD4 count was not an independent predictor of anti-TB drug induced hepatotoxicity.

Age was divided into ≤35 years and >35 years for the purpose of this analysis based on previous studies. Although, it has been reported that advanced age can be a risk factor for anti-TB drug induced hepatotoxicity [18], [28]–[30], in present study, no correlation was found between these age groups and the risk of developing anti-TB drugs induced hepatotoxicity. Also in other studies [16], [31], [32], advanced age was not risk for anti-TB drugs induced hepatotoxicity, a finding that is in consistent with the present study finding.

Although it has been reported that women are more predisposed to the risk of anti-TB drugs induced hepatotoxicity, this study did not find any correlation between gender and hepatotoxicity, a finding which is in agreement with study by Pukenyte E, et al. and Lima MFS, et al. [20], [21].

The article "Anti-Tuberculosis Drug Induced Hepatotoxicity among TB/HIV Co-Infected Patients at Jimma University Hospital, Ethiopia: Nested Case-Control Study" was published in 2013. Journal: PLoS One.

Use of ART has no significant association with the outcome, though it was considered to be a risk factor. This might be because considerable number of patients were on anti-TB drugs prior to the initiation of ART. Since most cases of hepatotoxicity occur in the first few weeks of treatment, ART will not be started for those patients of elevated liver enzyme. South African investigated whether serious adverse events during anti-TB therapy occur more frequently in HIV co-infected patients and concluded that severe adverse events occurrence was not related to ART [33]. Pukenyte E, et al. also reported no association between the concomitant initiation of ART and anti-TB drugs induced hepatotoxicity [20]. There could be also protective effect of ART as it improves clinical status and CD4 count of patients.

The use of cotrimoxazole has no effect on the development of hepatotoxicity. This might be because the majority of cases and controls were on cotrimoxazole preventive therapy. Similarly, there was no correlation between fluconazole use and anti-TB drugs induced hepatotoxicity.

Overall, the present study has limitation inherent in retrospective nested case-control analysis. Although, the nested case control study is a valid and efficient design, the sample evaluated by this study was smaller than the optimal sample size calculated for a full cohort case control study of this nature that might confer a low to moderate power to the present study. However, we used 3 controls for each case to increase power of efficiency. It is the suggestion of the present study to carry out multi-center population-based prospective cohort study of anti-TB drugs induced hepatotoxicity to provide data on the incidence, clinical features and its impact on TB treatment.

## Conclusions

Among TB/HIV co-infected patients, anti-TB drugs induced hepatotoxicity accounted for a considerable number of cases (11.5%). Most (93.9%) of hepatotoxicity incidents occurred in the intensive phase of treatment. Disseminated pulmonary TB and lower BMI were identified as independent predictors of occurrence of anti-TB drugs induced hepatotoxicity. Therefore, this study suggests that high risk patients to be identified prior to initiation of anti-TB drugs. The first 8 weeks is the critical period that requires vigilant monitoring of the toxicity indicators. Clinicians should recognize patients with disseminated pulmonary TB and lower BMI to monitor liver enzyme levels closely during the intensive phase of TB treatment of TB/HIV co-infected patients so as to ensure the best possible care. Therefore, more research and efforts are warranted in order to enhance the diagnosis and the prevention of anti-TB drugs induced hepatotoxicity.
